The article "Susceptibility Assessment of Multidrug Resistant Bacteria to Natural Products" was published in 2020. Journal: Dose Response.

# Susceptibility Assessment of Multidrug Resistant Bacteria to Natural Products

**DOI:** 10.1177/1559325820936189

**Published:** 2020-07-06

**Authors:** Essam Hassan Mohamed, Youssef Saeed Alghamdi, Salama Mostafa Abdel-Hafez, Mohamed Mohamed Soliman, Saad H. Alotaibi, Magdy Yassin Hassan, Nasr Al-Deen Hany, Hamada H. Amer

**Affiliations:** 1 Department of Biology, Turabah University College, Taif University, Saudi Arabia; 2 Department of Microbiology, Faculty of Veterinary Medicine, Zagazig University, Zagazig, Egypt; 3 Immunobiology and Immunopharmacology Unit, Animal Reproduction Research Institute, Giza, Egypt; 4 Clinical Laboratories Sciences, Turabah University College, Taif University, Turabah, Saudi Arabia; 5 Biochemistry Department, Faculty of Veterinary Medicine, Benha University, Benha, Egypt; 6 Chemistry Department, Turabah University College, Turabah, Taif University, Saudi Arabia; 7 Reproductive Disease Department, Animal Reproduction Research Institute, Giza, Egypt; 8 Microbiology Laboratory, King Faisal Medical Complex, Saudi Arabia; 9 Animal Medicine and Infectious Diseases Department, Faculty of Veterinary Medicine, University of Sadat City, Egypt

**Keywords:** quercetin, acacia, clove, scanning electron microscope, DNA fragmentation, multiresistant bacteria

## Abstract

**Objective:**

The aim of this study was to examine the effect of some natural compounds against multidrug-resistant bacteria.

**Methods:**

Forty-three bacterial strains were collected. Disc diffusion and minimum inhibitory concentration (MIC) tests were carried out for natural compounds including quercetin, *Acacia nilotica*, *Syzygium aromaticum*, and *Holothuria atra*. Scanning electron microscope analysis and bacterial DNA apoptosis assays were performed.

**Results:**

*Staphylococcus aureus* strains were resistant to imipenim, ampicillin, and penicillin. Most *Escherichia coli* strains were resistant to amoxicillin, clavulanat, and ampicillin. Finally, tigecycline was effective with *Klebsiella pneumoniae* and was resistant to all antibiotics. Only *S aromaticum* had an antibacterial effect on *K pneumoniae*. Most *S aureus* strains were sensitive to *S aromaticum*, *A nilotica*, and quercetin. All examined natural extracts had no effect on *E coli*. *Holothuria atra* had no effect on any of the strains tested. Minimum inhibitory concentration and minimum bactericidal concentration values for examined plants against *S aureus* were 6.25 to 12, 1.6 to 3.2, and 9.12 to 18.24 mg/mL, respectively. *Syzygium aromaticum* was active against *K pneumoniae* with an MIC of 12.5 mg/mL. Scanning electron microscope analysis performed after 24 and 48 hours of incubation showed bacterial strains with distorted shapes and severe cell wall damage. *Syzygium aromaticum*, quercetin, and *A nilotica* showed clear fragmentations of *S aureus* DNA.

**Conclusions:**

Current findings confirmed the beneficial effect of using natural products such as *clove (S aromaticum)*, quercetin, and *A nilotica* as a promising therapy to overcome multidrug resistant bacteria.

## Introduction

Bacterial resistance is one of the most critical problems currently facing public health agencies worldwide. Both human and veterinary medical practices use a large variety of antibiotics; unfortunately, bacterial resistance has seriously lowered their efficacy.^1^ Bacterial resistance may occur naturally, but the long history of the misuse of antibiotics in the treatment of viral and other diseases not caused by bacteria has accelerated the occurrence of bacterial resistance. Increased resistance is becoming problematic to treat as antibiotics become ineffective.^2^ Recent research has examined how to change the way antibiotics are prescribed and used. One goal of pharmaceutical companies is the discovery of new substances to reduce and treat bacterial resistance. Natural extracts are one of the alternative sources available that may solve the problem of bacterial resistance.

Multiple drug resistance has increased because of the random use of antibiotics in the treatment of infectious diseases,^3,4^ a critical situation that has forced researchers to seek new antimicrobial substances. Natural extracts are considered to be one of the major natural sources containing as yet undiscovered antimicrobial substances.^5^ Therefore, there is a need to develop alternative ways to treat infectious diseases using medicinal plants^6,7^ and substances secreted by some animals, such as sea cucumber (*Holothuria atra)*, a marine invertebrate found on the seafloor.^8^ *Holothuria atra* has cytotoxic, antioxidant, antibacterial, anti-inflammatory, antiviral, antitumor, and anticancer properties.^9^ Clove (*Syzygium aromaticum*) has been used in traditional medicine for thousands of years in Europe and Asia.^10^ Clove oil has a great many medicinal uses, with anti-inflammatory, anti-mutagenic, and antioxidant properties. It has also been used as an antibiotic because of its antimicrobial properties. Many people use cloves and clove oil in alternative remedies and the treatment of many infections.^11,12^ *Acacia nilotica* is a plant with a variety of functions that can be used in the treatment of many diseases.^13^ It contains several bioactive components,^14^ including phlobatannin, tannin, gallic acid, catechin, protocatechuic acid, pyrocatechol, epigallocatechin, 5-epigallocatechin-7gallate, and 7-digallate.^15^ The bark of the plant is commonly used for treatment of respiratory manifestations, diarrhea, leukoderma, and bleeding.^16^ Moreover, its tender leaves and pods are used in the treatment of *Klebsiella* sp., *Pseudomonas* sp., and *Salmonella typhimurium* infections in humans.^17^ Quercetin is a well-known bioflavonoid that has biological properties. It has beneficial antioxidant, anti-inflammatory, antimutagenic, anticancer, antimicrobial, and antiviral activities.^18^ The aim of this research was to study the antibacterial effects of some natural extracts and quercetin in a trial to treat and control some of the multidrug resistant bacteria considered dangerous to human and animal health.

## Methods

### Bacterial Samples

Forty-three different bacterial strains were included in this study: *Staphylococcus aureus* (n = 21), *Escherichia coli* (n = 17), and *Klebsiella pneumoniae* (n = 5). All bacterial strains were kindly donated by patients admitted to microbiological investigations at the King Faisal Hospital laboratories. All patients read, agreed to, and signed the ethical approval obtained from the Directorate of Health Affairs in Taif, Kingdom of Saudi Arabia. The original specimens (wounds, sputum, urine, catheters, and blood) were cultured on blood agar and MacConkey agar (Difco), then Gram staining was done, and complete diagnosis along with sensitivity test for all bacterial strains was done by Phoenix Automated Microbiology System (BD Diagnostics System). Each strain was freshly cultivated separately in tryptic soy broth (Difco) at 37 °C for 24 hours. The cells were harvested by centrifugation at 5000 × *g* for 10 minutes, washed twice, and then suspended to a final cell density equal to 0.5 McFarland turbidity standards (1.6 × 107 CFU/mL) just before the beginning of the experiment.

## Preparation of Natural Extracts

### Clove Water Extract

Clove (*S aromaticum)* flower buds were selected based on their traditional usage as folk medicine in our Arabic area. The plants were purchased in dried form from Ubuy Co. *Syzygium aromaticum* flower buds (10 g) were soaked in 100 mL cold, sterile distilled water for 24 hours. This clove–water mixture was incubated for 30 minutes in a water bath at 37 °C with frequent shaking and kept for another 24 hours.^19^

### Acacia nilotica Extract

*Acacia nilotica* seeds were purchased from Ubuy Co in dried form. Seeds were rinsed and dried at 28 °C ± 2 °C for 2 weeks. The seeds were minced using a blender. The powdered seeds (100 g) were soaked in 800 mL sterile distilled water with reflux for 6 hours. The resulting mixture was filtered and allowed to evaporate using a rotary evaporator at 50 °C. The dried extract was kept sterile and stored at −20°C until use.^20^ The identity of clove and *A nilotica* were confirmed by a botanist (Prof Yassin Al-ssodany) at the Botany Department, College of Science, Kafrelsheikh University, Egypt.

### Holothuria Atra

*Holothuria atra* were obtained from Thuwal. The taxonomy of *H atra* was confirmed according to the methods used in previous studies.^21^ The animals were transported in an ice box, rinsed thoroughly, and then the animal’s body wall was removed and soaked in a methanol water (50:50) solution for 16 hours with shaking. The mixture was filtered, and the remaining filtrate soaked in the 50:50 methanol water solution again. The 2 portions were pooled and concentrated using a rotary evaporator. The powdered extract was obtained by freeze drying and stored at −20 °C until use.^22^

### Quercetin

Quercetin was purchased from Sigma-Aldrich and freshly dissolved in dimethyl sulfoxide (DMSO) at a concentration of 200 mg/mL of DMSO just before the beginning of the experiment.

### Antibacterial Activity of Syzygium aromaticum, Acacia nilotica, Quercitin, and Holothuria atra

The antibacterial activity of *S aromaticum*, *A nilotica*, quercitin, and *H atra* was assessed using the method described by Duraipandiyan et al^23^ with slight modifications. Briefly, the bacterial count of each isolate used was adjusted to 0.5 McFarland turbidity standards in sterile saline, poured on the surface of a Petri dish containing Mueller Hinton agar (Difco), and properly spread. A volume of 50 µL of each of the stock concentrations of quercetin and *H atra* in DMSO (200 mg/mL), *A nilotica* (100 mg/mL distilled water), and *S aromaticum* (200 mg/mL, distilled water) was loaded on 6-mm sterile discs. An amoxicillin disc (10 µg/mL) and a ciprofloxacin disc (5 µg/mL) were used as negative and positive controls for the inhibition zones, respectively. The plates were incubated at 37 °C for 24 hours. The results represent the measurements of the inhibition zones. All experiments were repeated in triplicate.

### Determination of Minimum Inhibitory Concentration

The microdilution technique was used to determine the minimum inhibitory concentration (MIC) of *S aromaticum,* quercetin, and *A nilotica* as recommended by CLSI.^24^ With slight modifications, stock concentrations of *S aromaticum*, quercetin, and *A nilotica* were prepared. Each well was filled with 100 µL of Mueller Hinton broth (Difco) and 100 µL of each of the stock concentration of the 2 extracts; quercetin was added to the first well with a double-fold serial dilution. A volume of 100 µL of inoculated broth culture containing (1.6 × 107) CFU/mL was added to all wells except for negative control wells. Finally, the plates were incubated at 37 °C overnight. Wells containing DMSO in Mueller Hinton broth along with standardized bacterial inocula were used as growth control, while wells containing Mueller Hinton broth without any treatment or bacterial inoculum were used as negative control. The last well showing no visible turbidity provided the MIC value; wells showing no growth on nutrient agar after 24 hours of incubation provided the minimum bactericidal concentration (MBC) value.

### Scanning Electron Microscope

*Staphylococcus aureus* was cultured overnight in tryptic soy broth (Hi media), and the broth turbidity was adjusted to 0.5 McFarland turbidity standards and then treated with equal volumes of *S aromaticum,* quercetin, and *A nilotica* (MIC dose as in Table 1) and incubated for 24 and 48 hours to check the bacterial morphology using scanning electron microscope (SEM). The treated broth culture was fixed overnight with an equal volume of 2% glutaraldehyde in 5% sucrose. The specimens were prepared for scanning electron microscopy as described previously.^25^ The morphological changes were photographed under the analytical SEM (model JEOLJSM-6390 LA serial number PM14400099) in the Electron Microscope Unit of Taif University.

**Table 1.** Minimum inhibitory concentration (MIC) and MBC Tests of *Syzygium Aromaticum*, *Acacia nilotica, and* Quercetin Against the Bacterial Strains Examined.

Bacterial species	Broth microdilution method, MIC/MBC, mg/mL		
	*Syzygium aromaticum*	*Acacia nilotica*	Quercetin
*Staphylococcus aureus*	6.25/12	1.6/3.2	9.12/18.24
*Escherichia coli*	NT	NT	NT
*Klebsiella pneumoniae*	12.5/25	NT	NT

Abbreviations: MIC, minimum inhibitory concentration; MBC, minimum bactericidal concentration; NT, not tested.

### Bacterial Apoptosis

*Staphylococcus aureus* was grown in tryptic soy broth overnight at 37 °C, and the bacterial count was adjusted to 0.5 McFarland turbidity standards. A DNA cleavage assay was performed according to methods of Nagata^26^ with some modifications. The broth-cultured bacteria were incubated with an MIC dose of *S aromaticum,* quercetin, and *A nilotica* as shown in Table 1 and incubated at 37 °C for 8, 24, 48, and 72 hours for both *S aromaticum* and *A nilotica* and for 24, 48, and 72 hours for quercetin. Bacterial broth was precipitated after centrifugation at 10 000 RPM for 5 minutes. The bacterial pellets were suspended in 400 µL diethyl pyrocarbonate (DEPC) water and heated at 100 °C for 10 minutes, followed by centrifugation for 10 minutes at 20 000 × *g*. The clear supernatant was removed and saved for DNA precipitation and concentration. Ice-cold ethanol (1 mL) was added to the supernatant, shaken gently, and incubated at −20 °C overnight. The next day, it was centrifuged at 12 000 RPM for 10 minutes at 4 °C and the washed DNA pellets were left to air dry. The pellets were reconstituted by the addition of 100 µL nano pure water. The DNA concentration was measured using a BIO-RAD spectrophotometer at OD 260. Extracted DNA (250 ng) was loaded in a 1% agarose gel stained with ethidium bromide and imaged using a gel documentation system (Bio-Rad).

## Results

### Antibiotic Sensitivity Test

The multidrug resistant bacterial strains collected for this study are *S aureus, E coli,* and *K pneumoniae*. Strains were collected from wounds, sputum, urine, catheters, and blood. The collected strains were tested against different antibiotics using The Phoenix Automated Microbiology System. The results of antibiograms showed that the most effective drug against *S aureus* were daptomycin, linezolid, moxifloxacin, and vancomycin (100%). In contrast, all *S aureus* strains were resistant to imipenim, penicillin, and ampicillin (100%, 95.2%, and 95.2%, respectively) as seen in Figure 1. *Escherichia coli* was sensitive to amikacin (94%) and resistant to amoxicillin, clavulanat, and ampicillin with approximate percentage of 94% as seen in Figure 2. *Klebsiella pneumoniae* was slightly sensitive to tigecycline and resistant to all tested antibiotics (Figure 3).

**Figure 1.** Antibiotic sensitivity test for *Staphylococcus aureus* strains (n = 21). R; resistant, S; sensitive. The most effective drug were daptomycin, linezolid, moxifloxacin, and vancomycin (100%). Meanwhile, all strains were very resistant to imipenim, penicillin, and ampicillin (100%, 95.2%, and 95.2%, respectively).

**Figure 2.** Antibiotic sensitivity test for *Escherichia coli* (n = 17). R; resistant, S; sensitive. All *E coli* strains were sensitive to amikacin (94%). All strains were resistant to amoxicillin, clavulanat, and ampicillin (94%).

**Figure 3.** Antibiotic sensitivity test for *Klebsiella pneumoniae* strains (n = 5). R; resistant, S; sensitive. All *Klebsiella pneumoniae* strains were slightly sensitive to tigecycline and were resistant to all tested antibiotics.

### Disc Diffusion Test of Syzygium aromaticum, Quercetin, Acacia nilotica, and Holothuria atra

Next, we examined the antibacterial activity of *S aromaticum,* quercetin, *A nilotica,* and *H atra* against bacterial strains using the disc diffusion test. The results of the antimicrobial tests are shown in Table 2. The highest inhibition zone was achieved with *S aromaticum*, followed by quercetin and *A nilotica,* with zone sizes of 18.14 ± 0.659, 16.95 ± 0.760, and 14.94 ± 0.368 mm, respectively. Only *S aromaticum* demonstrated antibacterial activity against *K pneumoniae,* with an inhibition zone size of 13.76 ± 0.545 mm. None of the natural extracts examined had any effect on any of the *E coli* tested, as shown in Figure 4. Finally, the extract of *H atra* was not effective against any of the bacterial strains tested.

**Table 2.** Inhibitory Activity of *Syzygium aromaticum, Acacia nilotica,* and Quercetin Using the Disc Diffusion Test.^a^

Inhibition zone in mm, mean ± SE					
	*Syzygium aromaticum*	*Acacia nilotica*	Quercetin	*Holothuria atra*	Ciprofloxacin
*Staphylococcus aureus* (n = 21)	18.14 ± 0.659	14.94 ± 0.368	16.95 ± 0.760	Nz	20.33 ± 0.952
*Klebsiella pneumoniae* (n = 5)	13.76 ± 0.545	Nz	Nz	Nz	19.35 ± 0.969
*Escherichia coli* (n = 17)	Nz	Nz	Nz	Nz	18.71 ± 0.662

Abbreviations: Nz, no inhibition zone; SE, standard error.

^a^ Values are means ± standard error of means for 3 different experiments carried out in triplicate.

**Figure 4.** Disc diffusion test showing inhibition zones in mm. A, Inhibition zones of *Acacia nilotica*, ciprofloxacin, and amoxicillin. B, Inhibition zones of *Syzygium aromaticum*, ciprofloxacin, and amoxicillin. C, Inhibition zones of quercetin, ciprofloxacin, and amoxicillin.

Minimum inhibitory concentration and MBC test results are shown in Table 1. The results showed that the MIC/MBC of *S aromaticum*, quercetin, and *A nilotica* were 6.25/12.5 mg/mL, 9.12/18.24 mg/mL, and 1.6/3.2mg/mL, respectively, against *S aureus* strains. *Syzygium aromaticum* extract was the most effective product against *K pneumoniae,* with MIC/MBC values of 12.25/25 mg/mL, as show in Table 1.

### Scanning Electron Microscopy

Scanning electron microscopy of the staphylococcal strains after incubation with *S aromaticum*, quercetin, and *A nilotica* at the MIC dose for 24 and 48 hours is shown in Figures 5 and 6. The results of SEM revealed that *S aromaticum*, *A nilotica*, and quercetin induced a significant variation in the size of the bacterial cells compared to those of controls (Figures 5 and 6). After 24 hours of incubation, the cells became smaller compared to those of control untreated bacteria (Figure 5A and B and Figure 6A). After 48 hours of incubation, the changes in the bacterial morphology became clearer, with distorted shapes compared to those of untreated controls. These changes resulted from the deformity of the bacterial cell wall with a change in the round characteristic shape of the bacterium. In addition, there were clear areas with no bacterial growth as seen in Figure 5B and D and Figure 6B.

**Figure 5.** Scanning electron microscope (SEM) analysis. (A) *Syzygium aromaticum* with *Staphylococcus aureus* after 24 hours. (B) *Syzygium aromaticum* with *S aureus* after 24 hours; (C) *Acacia nilotica* with *S aureus* after 24 hours; (D) *Acacia nilotica* with *S aureus* after 48 hours.

**Figure 6.** A, Quercetin with *Staphylococcus aureus* after 24 hours. B, Quercetin with *Staphylococcus aureus* after 48 hours. C, Normal control.

### Bacterial Apoptosis

DNA fragmentation of quercetin, *A nilotica,* and *S aromaticum* was performed using the bacterial apopotosis technique. As shown in Figures 7 and 8, incubation of *S aureus* in tryptic soy broth with quercetin (9.12 mg/mL) for 24, 48, and 72 hours completely induced 100% DNA cleavage in time dependent manner. Bacterial DNA did not appear in an ethidium bromide stained gel (1%) when compared to the control lane (*S aureus* without treatment). In parallel analyses, DNA cleavage was assessed after incubation with *A nilotica* and *S aromaticum*. Lanes 3 to 6 and 9 to 12 for *A nilotica* and *S aromaticum,* respectively, show bacterial DNA cleavage as a white smear and white illumination starting from 8 hours of incubation through 72 hours after treatment when compared with lanes 2 and 8 (untreated bacteria; Figure 8). DNA was fragmented and degraded in time-dependent manner confirming antibacterial activity for *A nilotica* and *S aromaticum*.

**Figure 7.** DNA cleavage of quercetin with *Staphylococcus aureus*. Lane 1: DNA ladder; Lane 2: *S aureus* control without treatment; Lane 3: quercetin at 24 hours; Lane 4: quercetin at 48 hours; and Lane 5: quercetin at 72 hours.

**Figure 8.** DNA cleavage of *Acacia nilotica* and *Syzygium aromaticum* with *Staphylococcus aureus*. Lane 1: 100-bp DNA ladder; Lane 2: *Staphylococcus aureus* control without treatment; Lanes 3-6: *Acacia nilotica* treated bacteria for 8, 24, 48, and 72 hours; Lane 7: 100 DNA ladder; Lane 8: *S aureus* control without treatment; Lanes 9-12: *Syzygium aromaticum* treated bacteria for 8, 24, 48, and 72 hours.

## Discussion

The appearance of multidrug resistant pathogens threatens the clinical effectiveness of many commonly used antibiotics.^27^ As a result, there is an increasing demand for the discovery of new antibiotics with novel modes of action against these multidrug resistant pathogens. Antimicrobial substances of natural origin have the potential to play a great therapeutic role in the control of numerous infectious diseases.^28^ Antimicrobial testing of *S aureus, E coli,* and *K pneumoniae* revealed that the most effective drug against *S aureus* were linezolid, daptomycin, moxifloxacin, and vancomycin (100% sensitive). Meanwhile, they were all resistant to imipenim, ampicillin, and penicillin (100%, 95.2%, and 95.2%, respectively). Previous studies that examined the antibiotic susceptibility of *S aureus* reported high rates of resistance to penicillin (98.9%) and erythromycin (61.6%), with only 1 isolate resistant to vancomycin.^29^ *Escherichia coli* strains were sensitive to amikacin and ceftazidime (94% and 88%, respectively) and were resistant to amoxicillin, clavulanat, and ampicillin (94%). Finally, *K pneumoniae* strains were sensitive to tigecycline and resistant to all tested antibiotics. Comparable results reported by Gautam et al^30^ confirmed that *E coli* strains were sensitive to ceftazidime (99%) and imipenem (83%). *Klebsiella pneumoniae* was sensitive to cefotaxime (87%). Using disc diffusion techniques, MIC and MBC tests were performed to detect any antimicrobial actions of natural extracts and quercetin. The aqueous extract of *S aromaticum* was the most effective against *S aureus* strains, with a mean zone size of 18.14 ± 0.659 mm; additionally, it was the only product tested in this study shown to be effective against *K pneumoniae,* with a mean zone size of 13.76 ± 0.545 mm. No inhibition zones were observed following tests with any of the *E coli*. The MIC value was 6.25 and 12.5 mg/mL for *S aureus* and *K pneumoniae*, respectively. Other studies carried out in parallel investigated the effect of *S aromaticum* against several gram-positive and gram-negative bacteria. The MIC values for *S aureus* and *E coli* were 5.4 ± 1.08 mg/mL; the inhibition zones were 25.3 ± 0.66 and 31.6 ± 0.88 mm. This expected effect was attributed to the chemical compounds known as eugenol, caryophyllyne, and eugenyl acetate.^31^ While others^32^ have shown that the ethanolic extract of *S aromaticum* inhibited the growth of food borne pathogens such as *S aureus* and *K pneumoniae*, which contradicts our findings regarding a lack of activity against *E coli,* it is possible that this could be attributed to the method of extraction used in both studies.

The aqueous extract of *A nilotica* showed strong suppression of clinical strains of *S aureus* with mean inhibition zones of 14.94 ± 0.368 mm. The MIC and MBC values were 1.6 and 3.2 mg/mL, respectively. Previous reports have confirmed that *A nilotica* was active against *S aureus*, *E coli,* and *K pneumoniae,* respectively. The MIC and MBC for *A nilotica* against *S aureus* were 0.5 and 1.0 mg/mL^33^ and against *E coli* were 6.25 and 12.5 mg/mL.^34^ As confirmed before, the antimicrobial activity of *A nilotica* extract is attributed to terpenes thought to cause membrane disruption due to lipophilic activity.^35^ It may be that the outer membrane layer of lipopolysaccharides in the cell wall of gram-negative bacteria is unique, rendering them impermeable to certain antibacterial agents and explaining why the effect is potent against gram-positive bacteria and weak against gram-negative strains.^36^ Other studies have attributed the antimicrobial effects of *A nilotica* to the methyl esters, methyl functional groups, and unsaturated furan ring it contains.^36^

Flavonoids, a group of chemicals present in plants and also known as phytonutrients, have a wide range of antimicrobial activities beneficial to humans. Previous studies of the antibacterial activity of flavonoids has demonstrated that they include inhibition of nucleic acid synthesis, inhibition of energy synthesis, reduction in cell attachment (biofilm formation), changes in cell permeability, and cytoplasmic membrane damage.^37^ Disc diffusion tests have shown that quercetin (a major flavonoid) strongly suppressed most strains of *S aureus,* with an inhibition zone of 16.95 ± 0.760 mm. The MIC and MBC values of quercetin were 9.12/18.24 mg/mL. Quercetin did not affect the gram-negative bacteria tested in this study. Quercetin was more effective against gram-positive bacteria. A previous study showed that quercetin disrupted cell walls and was effective against *S aureus* but not *E coli*.^38^

*Holothuria atra* extracts have been shown to have strong suppressive effects against bacterial and fungal pathogens. However, in this study, *H atra* exerted no effect on any of the bacterial strains tested. Similar results have been reported by others^39^ for *Candida albicans, Pseudomonas aeruginosa, and K pneumoniae*, but the extract has been reported to have an antibacterial effect against *Staphylococcus epidermidis*. The difference in results may be due the high fat content of the extract or a difference in extraction methods. Comparable studies showed that a methanolic extract of *H atra* had a potent antimicrobial effect against *Aspergillus niger*. However, another study using the same methanolic extract demonstrated no antibacterial effects against *C albicans, S aureus, P aeruginosa,* or *E coli*.^40^

Scanning electron microscope analysis was also included to investigate the mode of action of the natural extracts and quercetin compound examined. Past studies have reported that most of the treated bacterial cells became pitted, deformed, and broken, indicating that the *A nilotica* aqueous extract had a harmful effect on the cell wall of the bacteria strains examined.^41^ Other studies using field emission SEM reported that methanolic seed extracts of *S cumini* induced a significant variation in the size of *Bacillus subtilis* cells.^42^ Scanning electron microscope analysis of the effects of treatment with quercetin showed that it exhibited antibacterial activity characterized by disruption of the integrity of the cell walls in both gram-positive and gram-negative bacteria.^43^

A bacterial apoptosis technique was used to assess the mode of action of the products tested. *Syzygium aromaticum,* quercetin, and *A nilotica* induced lysis of and/or injury to bacterial DNA. Using MIC and Triplex PCR showed the time-dependent effects of these agents on bacterial DNA, with the most pronounced effects observed at 72 hours of incubation, confirmed by the absence of bacterial DNA on an ethidium bromide stained gel (1%). A previous study that examined aqueous extract of *S aromaticum* induced DNA fragmentation in *B subtilis* at 24, 48, and 72 hours of incubation reported time-dependent results^42^ that coincide with our findings. This indicates that the aqueous extract of *S aromaticum* has a pronounced effect on the degradation of DNA of *S aureus* accompanied by inhibition of bacterial protein synthesis.

## Conclusions

This study confirmed the antibacterial activity of *S aromaticum*, quercetin, and *A nilotica* against gram-negative and gram-positive bacteria. These observations can be exploited to treat bacterial infections using natural products instead of commonly used antibiotics or in combination with them.
